RETRACTED

# Upregulation of PTEN in Glioma Cells by Cord Blood Mesenchymal Stem Cells Inhibits Migration via Downregulation of the PI3K/Akt Pathway

**DOI:** 10.1371/journal.pone.0010350

**Published:** 2010-04-26

**Authors:** Venkata Ramesh Dasari, Kiranpreet Kaur, Kiran Kumar Velpula, Meena Gujrati, Daniel Fassett, Jeffrey D. Klopfenstein, Dzung H. Dinh, Jasti S. Rao

**Affiliations:** 1 Department of Cancer Biology and Pharmacology, University of Illinois College of Medicine at Peoria, Peoria, Illinois, United States of America; 2 Department of Pathology, University of Illinois College of Medicine at Peoria, Peoria, Illinois, United States of America; 3 Department of Neurosurgery, University of Illinois College of Medicine at Peoria, Peoria, Illinois, United States of America; The University of Chicago, United States of America

## Abstract

**Background:**

PTEN (phosphatase and tensin homologue deleted on chromosome ten) is a tumor suppressor gene implicated in a wide variety of human cancers, including glioblastoma. PTEN is a major negative regulator of the PI3K/Akt signaling pathway. Most human gliomas show high levels of activated Akt, whereas less than half of these tumors carry PTEN mutations or homozygous deletions. The unique ability of mesenchymal stem cells to track down tumor cells makes them as potential therapeutic agents. Based on this capability, new therapeutic approaches have been developed using mesenchymal stem cells to cure glioblastoma. However, molecular mechanisms of interactions between glioma cells and stem cells are still unknown.

**Methodology/Principal Findings:**

In order to study the mechanisms by which migration of glioma cells can be inhibited by the upregulation of the PTEN gene, we studied two glioma cell lines (SNB19 and U251) and two glioma xenograft cell lines (4910 and 5310) alone and in co-culture with human umbilical cord blood-derived mesenchymal stem cells (hUCBSC). Co-cultures of glioma cells showed increased expression of PTEN as evaluated by immunofluorescence and immunoblotting assays. Upregulation of PTEN gene is correlated with the downregulation of many genes including Akt, JUN, MAPK14, PDK2, PI3K, PTK2, RAS and RAF1 as revealed by cDNA microarray analysis. These results have been confirmed by reverse-transcription based PCR analysis of PTEN and Akt genes. Upregulation of PTEN resulted in the inhibition of migration capability of glioma cells under *in vitro* conditions. Also, wound healing capability of glioma cells was significantly inhibited in co-culture with hUCBSC. Under *in vivo* conditions, intracranial tumor growth was inhibited by hUCBSC in nude mice. Further, hUCBSC upregulated PTEN and decreased the levels of XIAP and Akt, which are responsible for the inhibition of tumor growth in the mouse brain.

RETRACTED

**Conclusions/Significance:**

Our studies indicated that upregulation of PTEN by hUCBSC in glioma cells and in the nude mice tumors downregulated Akt and PI3K signaling pathway molecules. This resulted in the inhibition of migration as well as wound healing property of the glioma cells. Taken together, our results suggest hUCBSC as a therapeutic agent in treating malignant gliomas.

## Introduction

Despite many advances in the treatment of malignant glioblastoma via surgery, radiotherapy and chemotherapy, patients afflicted with this disease continue to have a very poor prognosis [1]–[3]. Malignant glioblastoma is characterized by rapid cell proliferation, high invasion and genetic alterations [4]–[6]. A number of genetic alterations are involved in oncogenesis, including deactivation of tumor suppressor genes such as PTEN (phosphatase and tensin homologue deleted on chromosome ten) [7]. PTEN is a tumor suppressor gene implicated in a wide variety of human cancers and is a major negative regulator of the PI3K/Akt signaling pathway. Most human glioblastomas show high levels of activated Akt, whereas less than half carry PTEN mutations or homozygous deletions. There are several lines of evidence implicating PTEN in the regulation of cellular migration and invasion. It has also been suggested that PTEN may regulate cell migration by directly dephosphorylating FAK in the DBTRG-05MG glioblastoma cell line [8]. PTEN plays a significant role in inducing G_1_ cell cycle arrest and apoptosis, along with regulating cell adhesion, migration and differentiation [9], [10]. Dey *et al*. [11] studied glioma cell migration on vitronectin, which binds α_v_β_3_ integrin, and showed that PTEN's protein phosphatase activity negatively regulated RAC1 indirectly by regulating the activity of the SRC-family kinase, FYN. Recent insights into the biology of gliomas include the finding that tyrosine kinase receptors and signal transduction pathways play a role in tumor initiation and maintenance [12]. PTEN is a tumor suppressor with phosphatase activity *in vitro* against both lipids and proteins and other potential non-enzymatic mechanisms of action. Davidson's recent data provides a novel tool to address the significance of PTEN's separable lipid and protein phosphatase activities and suggests that both activities suppress proliferation and both activities are required in concert to achieve efficient inhibition of invasion [13]. However, it is not clear whether PTEN genuinely regulates cell migration, tumor invasiveness and metastasis *in vivo* using the mechanisms and pathways defined by *in vitro* systems [14].

RETRACTED

Recent studies have indicated that mesenchymal stem cells (MSCs) have the capacity to target therapeutic genes to malignant glioma [15]–[17]. Human umbilical cord blood is a rich source of both hematopoietic stem cells and MSCs [18], [19]. Stem cells derived from umbilical cord show higher proliferation and expansion potential than adult bone marrow stem cells [20], [21]. Human umbilical cord-derived mesenchymal stem cells (hUCBSC) have been regarded as an alternative cell source for cell transplantation and cell therapy because of their hematopoietic and non-hematopoietic (mesenchymal) potential [19], [22], [23].

To study the mechanisms by which migration of glioma cells can be inhibited by the upregulation of PTEN gene, we used two glioma cell lines (SNB19 and U251) and two glioma xenograft cell lines (4910 and 5310) alone and in co-culture with hUCBSC. We evaluated whether hUCBSC are capable of inhibiting the migration capability of glioma cells both *in vitro* and *in vivo*, and whether this effect is mediated by downregulation of the PI3K-Akt pathway.

## Results

### Co-culture of glioma cells with hUCBSC upregulates PTEN

For all the experiments of this study, we used hUCBSC which are positive for CD29 and CD81, as confirmed by immunocytochemistryand FACS analyses (data not shown). To evaluate the efficiency of hUCBSC, we tested the effect of hUCBSC on glioma cells in co-cultures. All of the four glioma cell lines of the present study were co-cultured with hUCBSC for 3 days and the total RNA was extracted and reverse-transcribed to cDNA. We ran cDNA microarrays for PI3K-Akt pathway as described in Materials and Methods. We found that PTEN is upregulated many times over in the four tested cell lines. Many genes related to PI3K-Akt pathway were downregulated in SNB19, U251 and 4910 cells, whereas most of the genes in 5310 cells were brought down to normal levels. The upregulation of PTEN gene was correlated with the downregulation of numerous genes including Akt, JUN, MAPK14, PDK2, PI3K, PTK2, RAS and RAF1 as revealed by cDNA microarrays (Table 1). To check for PTEN expression levels, we carried out immunofluorescence assays with the PTEN antibody and found that with hUCBSC treatment, significant upregulation of PTEN took place in all of the glioma cells in the present study (Fig. 1A). This indicates that hUCBSC upregulated PTEN in glioma cells. To confirm these results, we checked the expression of PTEN, Akt and PI3K at both the transcriptional and translational levels. In both cases, PTEN was upregulated in hUCBSC-treated cancer cells whereas Akt, phospho-Akt and PI3K were downregulated as compared to control cells (Figs. 1B and 1C). To evaluate whether hUCBSC undergo any changes after co-culturing with glioma cells, hUCBSC were grown in conditioned media of glioma cells and observed for changes in PTEN expression at both transcriptional and translational levels. We did not observe any significant changes in the levels of PTEN in hUCBSC grown in glioma conditioned media (Figs. 1D and 1E). These results confirm that hUCBSC upregulates PTEN in glioma cells and shows a negative effect on PI3K and Akt levels as well as the phosphorylation status of the Akt^Ser473^ molecules.

RETRACTED

**Figure 1:** Upregulation of PTEN in hUCBSC-treated co-cultures of glioma cells. (A) Fluorescent microscopic images demonstrate PTEN expression (red fluorescence). SNB19, U251, 4910 and 5310 cells were co-cultured with hUCBSC for 3 days and processed for immunofluorescence. Immunostaining was performed with Alexa flour-594 conjugated PTEN antibodies. All sections were stained with DAPI to show nuclear localization. Insets show DAPI. n ≥ 3. Scale bar  = 100 µm. (B) Equal amounts of protein (40 µg) from single cultures and co-cultures were loaded onto 12% SDS gels and transferred onto nitrocellulose membranes, which were then probed with respective antibodies. GAPDH was used as a positive loading control. (C) Reverse transcription-based PCR analysis of PTEN, Akt and PI3K in co-cultures. β-actin was used as a positive loading control. Each blot and gel is representative of experiments performed in duplicate with each sample (n = 3). hUCBSC were grown in conditioned media from hUCBSC (control), SNB19, U251, 4910 and 5310 conditioned media for 3 days and the lysates (80 µg for each lane) were subjected to (D) Western analysis for PTEN or (E) Reverse-transcription based PCR analysis. CM =  conditioned medium.

**Table 1:** Effect of hUCBSC on glioma cells after co-culture (cDNA microarray results of PI3K-AKT pathway).

Gene	Description	Fold up or down regulation SNB19 U251 5310 4910			
AKT1/PKB	V-akt murine thymoma viral oncogene homolog 1	**−4.53**	**−2.35**	**−1.12**	**−4.00**
FOXO1	Forkhead box O1	**−3.43**	**−3.81**	**1.03**	**−6.96**
JUN	Jun oncogene	**−18.13**	**−3.10**	**−2.01**	**−13.93**
MAPK14	Mitogen-activated protein kinase 14	**−1.72**	**−3.32**	**−1.69**	**−10.56**
P110 (PIK3CA)	Phosphoinositide-3-kinase, catalytic, alpha polypeptide	**−7.89**	**1.77**	**1.14**	**−6.06**
P27, KIP I (CDKN1B)	Cyclin-dependent kinase inhibitor 1B (p27, Kip1)	**−4.23**	**−1.30**	**1.45**	**−10.56**
PAK1	P21 protein (Cdc42/Rac)-activated kinase 1	**−38.85**	**−3.43**	**1.06**	**−13.00**
PDGFRA	Platelet-derived growth factor receptor, alpha polypeptide	**1.09**	**−5.39**	**−1.08**	**1.52**
PDK2	Pyruvate dehydrogenase kinase, isozyme 2	**−41.64**	**−10.06**	**−1.47**	**−48.50**
PI3K (PIK3CG)	Phosphoinositide-3-kinase, catalytic, gamma polypeptide	**−6.87**	**−1.26**	**1.61**	**−4.29**
PIK3R2	Phosphoinositide-3-kinase, regulatory subunit 2 (beta)	**−13.74**	**−4.08**	**1.67**	**−22.63**
PTEN	Phosphatase and tensin homolog	**7.06**	**2.17**	**2.13**	**3.73**
PTK2	PTK2 protein tyrosine kinase 2	**−11.16**	**−2.35**	**−1.01**	**−16.00**
RAS (RASA1)	RAS p21 protein activator (GTPase activating protein) 1	**−19.43**	**−1.66**	**1.36**	**−5.66**
RAF1	V-raf-1 murine leukemia viral oncogene homolog 1	**−15.78**	**−5.98**	**−2.08**	**−4.00**

Human PI3K-Akt PCR arrays (SA Biosciences) were run using cDNA from single and co-cultures of glioma cells with hUCBSC. Real time PCR was carried out and changes in gene expression were illustrated as a fold increase/decrease according to manufacturer's instructions. The cut-off induction determining expression was 2.0 or −2.0 fold changes. Genes that met these criteria were considered to be upregulated or downregulated.

RETRACTED

### Conditioned media from co-cultured glioma and hUCBSC inhibits spheroid migration

To determine the effects of PTEN upregulation in glioma cells, we performed the spheroid migration assay using conditioned media from co-cultured glioma and hUCBSC cells. The spheroid model is a three-dimensional cell culture system that more closely resembles the *in vivo* situation inside a tumor [24]. Spheroid growth reflects the proliferation of tumor cells, while the migration assay measures the ability of the cells organized in a three-dimensional structure to migrate and proliferate [25]. The cell migration away from the spheroid was monitored over a period of 24 h to 48 h by photographing the mid plane of the spheroids at intervals of 24 h with an inverted Olympus phase contrast microscope. In conditioned media of untreated glioma cells, the cells from spheroids started migrating as early as 24 h, whereas in conditioned media of co-cultures, spheroid migration was delayed significantly, even after 48 h (Fig. 2A). We observed that spheroid migration was significantly inhibited in 5310 cells (51.19%) followed by 4910 (47.86%), U251 (41.95%) and SNB19 (41.4%) cells (Fig. 2B). In order to prove that PTEN is responsible for the inhibition of spheroid migration, glioma cells were grown in conditioned media from single and co-cultures. Similar to co-culture cell lysates, glioma cells grown in conditioned media also showed upregulated PTEN (Fig. 2C). In another experiment, spheroids were transfected with siRNA to PTEN (siPTEN) and then grown in conditioned media from co-cultures. We did not observe any significant change in the inhibition of spheroid migration (Figs. S1A and S1B). These results prove that upregulation of PTEN in glioma cells by conditioned media from co-cultured glioma and hUCBSC cells inhibit spheroid migration.

RETRACTED

**Figure 2:** Conditioned medium from co-culture of glioma cells with hUCBSC inhibits spheroid migration. (A) SNB19, U251, 4910 and 5310 cells were cultured in 96-well low attachment plates at a concentration of 5×10^4^ cells, and spheroids were allowed to grow for 24 h at 37°C with shaking at 40–60 rpm. The spheroids were then transferred to 48-well plates and maintained for another 24–48 h in conditioned media from single cultures and co-cultures. Spheroid migration was analyzed using a phase-contrast microscope. Scale bar  = 1000 µm. (B) Quantitative analysis of spheroid migration from (A). Error bars indicate SEM. *p <0.05. **p <0.01. n = 3. (C) Immunoblot analysis of PTEN from glioma cells grown in their respective control conditioned media and co-culture conditioned media.

### Inhibition of the wound healing capacity of glioma cells by hUCBSC

Glioma cells, in general, have very good wound healing capacity. In order to evaluate the effect of hUCBSC on wound healing, we checked the wound healing capacity of glioma cells in single cultures and co-cultures with hUCBSC. A wound was made in a sub-confluent cell monolayer and cells were allowed to migrate into the cell-free area. The distance moved by the cells in control and co-cultured plates, respectively, was compared. The mobility of glioma cells was inhibited in co-cultures compared to single cultures. We observed that SNB19 and U251 cells repair their wounds in 8 h; 4910 cells heal in 9 h and 5310 cells heal in 7 h. In co-cultures, hUCBSC inhibited this wound healing capacity (Fig. 3A). The wound healing capacity is significantly inhibited in 4910 cells (63.75%) as compared to U251 (53.74%), 5310 (50.99%) and SNB19 (49.99%) cells (Fig. 3B). In order to confirm, whether inhibition of wound healing is by soluble factors present in the conditioned media of co-cultures or due to cell-to-cell contact between glioma cells and hUCBSC, we performed another experiment with conditioned media from single cultures and co-cultures. Compared to complete media, glioma cells took long time to repair the wounds in conditioned media. For example, in SNB19 cells wound healing was observed after 23 h in conditioned medium compared to 8 h in complete medium. Similarly, wound healing was complete after 24 h in U251, after 21 h in 4910 and after 22 h in 5310 cells. However, glioma cells grown in hUCBSC conditioned medium and co-cultured conditioned medium did not show any inhibition of wound healing (Fig. S2A and S2B). Overall, these results indicate that cell-to-cell contact between hUCBSC and glioma cells is necessary which significantly decreased wound healing capacity of glioma cells.

RETRACTED

**Figure 3:** Monolayer wound-induced migration assay. A line was scratched with a 200-µm plastic pipette tip in SNB19, U251, 5310 and 4910 cultures and co-cultures with hUCBSC. They were allowed to grow at 37°C in 5% CO_2_ atmosphere. Every three hours, cells that had migrated to the wounded areas were photographed under a microscope for quantification of cell migration. Images are representative of three separate experiments. Scale bar  = 500 µm. (B) Quantitative analysis of wound-induced migration assay from (A). The results are presented as mean ± SEM of three experiments done in duplicate. *p <0.05. **p <0.001.

### Upregulation of PTEN by hUCBSC treatment has an anti-tumor effect in U251 and 5310 glioma nude mice models

Our *in vitro* experiments have proved that co-culture with hUCBSC can efficiently inhibit glioma cell migration and wound healing capacity. Therefore, we further investigated the anti-tumor effect of these stem cells *in vivo* using U251 and 5310 cells in nude mice. After the mice were implanted with U251, 5310 and hUCBSC as described in Materials and Methods, the mice were observed for 21 days. At that point, tumor samples were taken, and paraffin-embedded sections were prepared for immunohistopathological examination. Hematoxylin and Eosin (H&E) staining of the *in vivo* sections clearly showed that the tumors in hUCBSC-treated mice were inhibited significantly and were one-third of the size of the tumors in control mice brains (Fig. 4A). U251 tumors were much bigger in size and more invasive than 5310 tumors. Next, we checked for the presence of hUCBSC in tumor areas of the brains of both control and hUCBSC-treated mice brain sections by immunofluorescence. In hUCBSC-treated mice brain tissue, the presence of hUCBSC as confirmed by mesenchymal stem cells markers CD29 and CD81, clearly establishes the fact that hUCBSC are responsible for tumor size reduction observed in the hUCBSC-treated brains (Figs. 4B and 4C). These CD29 and CD81 positive cells were observed in tumor regions only. We could not detect them in normal areas of the brains. Further, we evaluated PTEN expression in nude mice brain sections by colocalization studies using PTEN and CD81 antibodies. Nude mice brains treated with hUCBSC clearly show that PTEN was highly upregulated in hUCBSC-treated mice (Fig. 4C). CD81 was observed in hUCBSC-treated mice sections only and they were absent in control tumor sections. Colocalization of PTEN and CD81 in hUCBSC-treated mice confirms that the upregulation of PTEN was the result of presence of hUCBSC. It is plausible that hUCBSC not only upregulated PTEN in glioma cells which are in contact with them but also in surrounding glioma cells. We also evaluated whether upregulation of PTEN in mice brains had any effect on X-linked inhibitor of apoptosis protein (XIAP) levels in tumor brains. For this, we did DAB immunohistochemistry on both control tumor and stem cell-treated brains. Tumor brains show high levels of XIAP expression, whereas hUCBSC-treated brains show reduced levels of XIAP expression (Fig. 4D). This confirms that upregulation of PTEN in tumors significantly decreased the levels of XIAP as to induce the cellular death of the glioma cells.

RETRACTED

**Figure 4:** Inhibition of intracranial tumors by hUCBSC *in vivo*. (A) Nude mice with pre-established intracranial human glioma tumors (U251 or 5310) were treated with hUCBSC by intracranial injection (2.5×10^5^). Fourteen days after hUCBSC administration, the brains were harvested, sectioned, and stained with Hematoxylin and Eosin (n≥3). Inset pictures show higher magnification at scale bar  = 100 µm. (B) Characterization of hUCBSC in tumor areas in nude mice brain sections: Fourteen days after hUCBSC administration, the brains were harvested, sectioned and immunoprobed with mesenchymal stem cell markers CD29 and CD81 using Alexa flour-594 secondary antibody. (n ≥ 3). Scale bar  = 100 µm. (C) Upregulation of PTEN in nude mice: Mice brain sections were immunoprobed with PTEN and CD81 using appropriate fluorescence-conjugated secondary antibodies. Secondary antibodies used for PTEN and CD81 were: goat anti-mouse Alexa flour-594 for PTEN and donkey anti-goat Alexa Fluor 488 for CD81, respectively. Scale bar  = 100 µm. (D) Downregulation of XIAP in mice: Mice brain sections were probed with XIAP antibody by DAB immunohistochemistry and counterstained with DAPI. Scale bar  = 100 µm. Inset pictures show DAPI. (n  = >3).

Further, to understand the molecular mechanisms of PTEN-induced tumor regression, we evaluated the tissue lysates of both control tumor brains and hUCBSC-treated tumor brains by immunoblotting. Similar to the *in vitro* results, the expression levels of PTEN is upregulated, whereas Akt, p-Akt, FAK and XIAP in tumor specimens from hUCBSC-treated mice were prominently downregulated (Fig. 5A). Next, we assessed the mRNA expression of PTEN, XIAP, FAK and PDGFR. All of these genes were highly downregulated after the hUCBSC treatment with the upregulation of PTEN (Figs. 5C and 5D).

**Figure 5:** *In vivo* expression of PTEN and other signaling proteins. Equal amounts of protein (40 µg) from tissue lysates of untreated and treated mice brains were loaded onto 10–14% SDS gels and transferred onto nitrocellulose membranes, which were then probed with respective antibodies. GAPDH was used as a positive loading control. (A) PTEN, Akt, pAkt, FAK and XIAP proteins with respect to GAPDH. (B) Western blot analysis of PI3K pathway related proteins. (C) Reverse transcription-based PCR analysis of PTEN, XIAP, FAK and PDGFR in brain tissue lysates. Each blot or gel is representative of experiments performed in duplicate with each sample (n = 3). (D) Real-Time PCR analysis of FAK, PTEN, XIAP and PDGFR genes of *in vivo* samples. n = 3. Error bars indicate SEM. *p <0.05.

RETRACTED

Signaling through the PI3Ks is frequently activated in many human cancers, including glioblastoma, because of loss of PTEN. Deletion or loss of PTEN function leads to failure to convert PIP3 back to PIP2, resulting in the deregulation of PI3K in the absence of upstream signals from receptor tyrosine kinases. Hence, we determined to check the expression of proteins related to the PI3K/Akt pathway (e.g., PI3K, RhoA, RAC1, CDC42 and PDGFR). We found that all were downregulated in mice brains treated with hUCBSC (Fig. 5B), showing that PTEN upregulation is inhibiting the PI3K/Akt pathway, thereby regulating the growth of tumor cells. These results confirm the anti-tumor effect of hUCBSC *in vivo* and that tumor cell migration *in vivo* is efficiently regulated by hUCBSC.

## Discussion

Malignant glioblastoma is a highly invasive tumor of the central nervous system. Currently available therapies offer only limited benefit for patients with glioblastoma. As such, there is an immediate necessity to develop new therapeutic approaches and to better understand the molecular pathogenesis of glioblastoma. PTEN mediates many of its effects on proliferation, growth, survival and migration through its PtdIns(3,4,5)P3 lipid phosphatase activity, suppressing phosphoinositide 3-kinase (PI3K)-dependent signaling pathways [26]. Re-expression of PTEN in mammalian cells lacking the enzyme has been found to inhibit the motility of several lineages of such cells, including mouse embryo fibroblasts and tumor-derived cells of glial and prostate origin [8], [27], [28], although most of these studies have not addressed the mechanism of action of PTEN. In this study, we investigated the effects of hUCBSC on the effects of migration of glioma cells by upregulation of PTEN. We observed that the stem cells are able to upregulate PTEN simultaneously downregulating the PI3K/Akt pathway and inhibiting the growth and migration of the cancer cells.

The Akt signaling pathway is very important in glioblastoma multiforme (GBM) progression, and this pathway is activated in the majority of primary GBM samples [29], [30] as well as in xenografts derived from GBM tumor samples [31]. Akt represents a nodal point in cell signaling and can be activated by several upstream events, including epidermal growth factor receptor amplification or mutation, loss of PTEN, and PIK3CA mutation. As such, targeting this pathway may be able to block glioblastoma multiforme proliferation secondary to a variety of upstream etiologies [32]. We observed a similar rate of Akt pathway activation in all four GBM cell lines used in this study (Fig. 1). When these glioma cells are co-cultured with hUCBSC, upregulation of PTEN has been observed with concomitant downregulation of Akt and phosphorylated form of Akt.

RETRACTED

Phosphatidyl-inositol-3-kinase (PI3K) can phosphorylate and activate Akt while PI3K is negatively regulated by the tumor suppressor gene PTEN, which has been shown to be non-functional in 20 to 40% of GBM [33]–[36]. Akt is over-activated in many glioblastomas due to the loss of PTEN function [37], [38]. Akt regulates the function of numerous downstream signaling proteins involved in cell cycle, proliferation, apoptosis and invasion, which are all important to tumorigenesis [39]. Activated Akt deregulates cell growth by stabilization of cyclin D and promotion of the nuclear entry of MDM2, leading to the degradation of p53 [40]. Akt might also inhibit p21 expression through its phosphorylation and activation of MDM2 and subsequent downregulation of p53-mediated transcription of p21 [41], [42]. On the other hand, activated Akt exerts anti-apoptotic activity by phosphorylating and inactivating pro-apoptotic signaling proteins, such as BAD and caspase 9 [39], [43]. The involvement of Akt in diverse tumorigenic activities suggests that Akt activation alone might be sufficient to induce cancer [44]. Moreover, Akt activation may contribute to tumor invasion/metastasis by stimulating secretion of matrix metalloproteinases [45]. Therefore, dysregulation of the PI3K/Akt signaling pathway may play an important role in tumor development and progression.

In the present study, hUCBSC are able to upregulate PTEN under both *in vitro* and *in vivo* conditions. This upregulation of PTEN decreased the expression of Akt and its phosphorylated form pAkt. Also, hUCBSC treatment resulted in the downregulation of XIAP, which is highly upregulated in glioma cells, both *in vitro* and *in vivo*. This in turn resulted in the dysregulation of PI3K/Akt signaling pathway and ultimately inhibited the survival of glioma cells. In addition, hUCBSC treatment downregulated PDGFR and Akt genes at the transcriptional and translational levels, this resulted in the inhibition of glioma migration. In order to understand the anti-cancer effect of hUCBSC, we examined their effect on migration and wound healing capacity of glioma cells. Through our experiments, we confirmed that hUCBSC effect on glioma cells decreased the levels of phosphorylated Akt, which alters both cell migration and wound healing capacity. Tumor invasion requires both tumor cell migration and the degradation of the extracellular matrix [46]. Cell motility is one of the crucial points of metastasis which is necessary for the tumor cell to move through the matrix and enter the circulation so that it can travel to a distant site [47]. In our study, we demonstrated that hUCBSC significantly reduced the migration of glioma cells from the spheroids (Fig. 2). Wound-healing assays showed a slower wound-closure following co-culture with hUCBSC treatment, indicating decreased glioma cell motility (Fig. 3).

RETRACTED

In our studies, we observed that PTEN upregulation accompanied XIAP downregulation. Previous studies support a role for XIAP in negatively regulating PTEN content *in vitro* and *in vivo* [48]. Decrease of XIAP protein levels in colon cancer cells in response to the apoptosis-inducing agent mesalazine is accompanied, among others, by an increase of PTEN content [49]. Exposure of mice to the apoptosis-inducing agent rosiglitazone modestly upregulates PTEN protein levels in HCT116-XIAP^+/+^ cell-derived tumors but markedly increases PTEN content in HCT116-XIAP^−/−^ cell-derived tumors [50]. Recently, it was proposed that XIAP acts as an E3 ubiquitin ligase for PTEN and promotes Akt activity by regulating PTEN content and compartmentalization [48]. Akt is one of the anti-apoptotic factors that must be activated through phosphorylation. The phosphorylation of Akt has previously been shown to be promoted by XIAP, another anti-apoptotic protein dictating the fate of normal and cancer cells [51], [52]. Our results are in accordance with the previous reports that downregulation of XIAP did result in the downregulation of Akt and inhibition of glioma cell growth.

Activation of PI3K occurs commonly in cancers including glioblastoma, the most common primary brain tumor. Activation of PI3K is associated with increased metabolism, suggesting potential dependence of cancer cells on PI3K signaling, and raising the possibility that blockade of PI3K signaling in glioma should effectively kill these cells [53]. PTEN encodes a phosphatase that dephosphorylates phosphatidylinositol-3,4,5 triphosphate to convert it to phosphatidylinositol-4, 5 bisphosphate. Therefore, inactivation of PTEN leads to increased levels of phosphatidylinositol-3,4,5 triphosphate and increased Akt activation [33]. Conversely, restoration of PTEN leads to inhibition of Akt. Recently, it was reported that survival times were significantly reduced in patients whose tumors showed PI3K pathway activation [54]. In our study with hUCBSC, we observed that PTEN upregulation decreases levels of PI3K and its associated signaling molecules, along with increased Akt inactivation. This ultimately resulted in the regression of tumor growth in nude mice brains.

RETRACTED

There have been no reports regarding the possible mechanisms by which hUCBSC are capable of upregulating PTEN in glioma cells. In our *in vivo* studies we observed that CD81, a mesenchymal stem cell marker, is co-localized with PTEN in glioma regions of the brain. This suggests that hUCBSC are in contact with the glioma cells and are able to upregulate PTEN in glioma cells in their vicinity. These results support previous reports from our laboratory, which show that cell-to-cell contact between hUCBSC and glioma cells is necessary to induce apoptosis in glioma cells by hUCBSC (58). Taken together, our results demonstrate that PTEN is an important component of the PI3K/Akt signaling pathway. The growth retardation of glioblastoma cells treated with hUCBSC is not only due to the reduction in migration and wound healing capability, but also due to the downregulation of Akt and PI3K pathway-related genes. Targeting PTEN using hUCBSC may be an effective new strategy for the molecular therapy of human cancers.

## Materials and Methods

### Ethics Statement

After obtaining informed consent, human umbilical cord blood was collected from healthy volunteers according to a protocol approved by the Peoria Institutional Review Board, Peoria, IL, USA. The consent was written and approved. The approved protocol number is 06–014, dated December 10, 2009. The Institutional Animal Care and Use Committee of the University Of Illinois College Of Medicine at Peoria, Peoria, IL, USA approved all surgical interventions and post-operative animal care. The consent was written and approved. The approved protocol number is 851, dated November 20, 2009.

### Culture of glioma cell lines

Two high-grade human glioma cell lines (SNB19 and U251) and two xenograft cell lines (4910 and 5310) were used for this study. SNB19 and U251 cells lines were obtained from American Type Culture Collection (ATCC, Manassas, VA). Two xenograft cell lines (4910 and 5310) were kindly provided by Dr. David James at University of California, San Francisco. SNB19 and U251 cells were grown in Dulbecco's modified Eagle medium (DMEM) supplemented with 10% fetal bovine serum and 1% penicillin-streptomycin in a humidified atmosphere containing 5% CO_2_ at 37°C. Xenograft cell lines (4910 and 5310) were grown in RPMI1640 medium supplemented with 10% fetal bovine serum and 1% penicillin-streptomycin in a humidified atmosphere containing 5% CO_2_ at 37°C. For all the cells, medium was replaced every 2 days. In experiments with conditioned medium, medium was replaced every day.

RETRACTED

### Isolation and culture of hUCBSC

After obtaining informed consent, human umbilical cord blood was collected from healthy volunteers according to a protocol approved by the Peoria Institutional Review Board, Peoria, IL, USA. Human umbilical cord blood was enriched by sequential Ficoll density gradient purification. Next, we selected cells using CD29^+^ and CD81^+^ markers as described previously [55]. Briefly, the nucleated cells were suspended at a concentration of 1×10^6^/ µL in Mesencult medium (Stem cell Technologies, Vancouver, Canada) supplemented with 20% fetal bovine serum (FBS) (Hyclone, Logan, UT), 1% penicillin-streptomycin (Invitrogen, Carlsbad, CA) and plated in 100-mm culture dishes. The cells were incubated for three days and the non-adherent cells were removed with medium replacement. After the cultures reached confluency, the cells were lifted by incubation with 0.25% trypsin and 1 mM ethylene diamine tetraacetic acid (EDTA) at 37°C for 3 to 4 min. Cells were diluted at a ratio of 1∶3 and replated and cultured at 37°C in an incubator with a 5% CO_2_ atmosphere. For co-culture experiments, hUCBSC and glioma cells were cultured at a ratio of 1∶4. Co-cultures were grown in the medium in which single glioma cells were grown. For all the cells, medium was replaced every 2 days. In experiments with conditioned medium, medium was replaced every day.

### Spheroid migration assay

Spheroid migration was assayed as described previously [56] with some modifications. Spheroids of SNB19, U251, 5310 and 4910 cells were prepared by seeding a suspension of 5×10^4^ cells in their respective media on ultra low attachment 96-well plates and cultured until spheroid aggregates formed. Single glioma spheroids were placed in the center of each well of a 0.5% agarose-coated 48-well microplate and 200 µL of conditioned media of single cultures and co-cultures with hUCBSC was added to each well. Spheroids were incubated at 37°C for 48 h, after which the spheroids were fixed and stained with Hema-3 (Fisher Scientific, Pittsburgh, PA) and photographed. The migration of cells from spheroids to monolayers was quantified using a microscope calibrated with a stage and ocular micrometer and represented graphically.

### Transfection of siPTEN

The glioma cells were cultured as mentioned previously. siRNA to PTEN was obtained from Cell Signaling Technology (Danvers, MA). Cells at 60–70% confluency in 100 mm tissue culture plates were transfected with 100 nM of siPTEN and control siRNA using Fugene HD as per manufacturer's instructions (Roche, Indianapolis, IN). Following transfection, after 60–72 h depending on the cell line, cell lysates were assessed for expression levels of PTEN using western blot analysis as per standard protocols.

RETRACTED

### Wound healing assay

These experiments were done in either single and co-cultures in complete media or in conditioned media of single and co-cultures. Glioma cells (1×10^6^) were seeded in a 100-mm culture plate and then cultured to at least 95% confluence. In a similar fashion, glioma cells were co-cultured with hUCBSC. Monolayer cells were washed with their respective media and then scraped with a plastic 200 µL pipette tip and then placed back in a 37°C incubator. The “wounded” areas were photographed by phase contrast microscopy at various time points (0, 3, 6, 8, 9, 10, 12, 21, 22, 23 and 24 h after scraping) depending on the cell line. The relative migration distance was calculated by the following formula: the relative migration distance (%) = 100 (A–B)/A, where A is the width of cell wounds before incubation, and B is the width of cell wounds after incubation. Results are expressed as the mean ± SEM.

### Immunocytochemistry

Cultured hUCBSC were checked for mesenchymal markers by immunocytochemistry. Cultured cells plated in 2-well chamber slides were rinsed twice with phosphate buffered saline (PBS) and fixed in 4% paraformaldehyde. After additional PBS rinses, cells were blocked with 0.1 M PBS with 1% bovine serum albumin (BSA) for 1 h. Primary antibodies (1∶100 dilutions) specific for mesenchymal markers: mouse anti-CD29 (Millipore, Danvers, MA) and goat anti-CD81 (Santa Cruz Biotechnology, Santa Cruz, CA) and primary antibody specific for PTEN were diluted in goat serum and applied overnight at 4°C. Texas-Red conjugated anti-mouse or anti-goat secondary antibodies were diluted (1∶200) in goat serum and applied individually for 1 to 2 h at room temperature. Before mounting, the cells were stained with 4′, 6-diamidino-2-phenylindole (DAPI). The cells were observed using a fluorescence microscope (Olympus IX71, Olympus, Melville, NY) and/or a confocal microscope (Olympus Fluoview, Olympus, Melville, NY) and photographed.

### RNA extraction and quantitative real time PCR

All primer sequences were determined using established human GenBank sequences. Primer sequences were designed using Primer3 software (v.0.4.0). For real time polymerase chain reaction (RT-PCR) analysis and RT-PCR-based microarray analysis (RT^2^ Profiler PCR Array, SuperArray, Frederick, MD), total RNA was isolated from control and hUCBSC-treated cancer cells. Total cellular RNA was extracted using RNeasy kit (Qiagen, Valencia, CA), and RNA quality was determined by running a sample with RNA loading dye on a 1% agarose gel and checking for distinct 18S and 28S rRNA bands, indicating lack of degradation. Quantity of RNA was determined by A_260_ measurement. We used RNA whose A_260_∶A_280_ ratio is greater than 2.0. Samples were either used immediately or frozen at −80°C until use in RT-PCR. Total RNA was reverse transcribed into first strand cDNA using Transcriptor First Strand cDNA Synthesis Kit (Roche, Indianapolis, IN). Each cDNA was tested by running PCR using GAPDH and β-actin primers as a control for assessing PCR efficiency and for subsequent analysis by 2% agarose gel electrophoresis. PCR amplification was performed using the primer sets, amplified by 35 cycles (94°C, 1 min; 60°C, 1 min; 72°C, 1 min) of PCR using 20 pM of specific primers. Further quantitative analysis of genes was done by SYBR green based real-time PCR using Bio-Rad iCycler iQ Real-Time PCR Detection System. Each sample was measured in triplicate and normalized to the reference GAPDH or β-actin gene expression. The value of each well was determined and the average of the three wells of each sample was calculated. For samples that showed no expression of the test gene, the value of minimum expression was used for statistical analysis. Delta C_T_ (ΔC_T_) and ΔΔC_T_ values were calculated and the fold change in the test gene expression was finally calculated. A statistical evaluation of real-time PCR results was performed using one-way analysis of variance (ANOVA) to compare test gene expression between cancer cells and their co-cultures with hUCBSC.

RETRACTED

### Primers used for PCR

FAK Sense 5′ggtgcaatggagcgagtatt3′

Antisense 5′gccagtgaacctcctctga3′

PTEN Sense 5′ccaggaccagaggaaacct3′

Antisense 5′gctagcctctggatttga3′

Akt Sense 5′catcacaccacctgaccaa3′

Antisense 5′ctcaaatgcacccgagaaat3′

PI3K Sense 5′cccctccatcaacttcttca3′

Antisense 5′cggttgcctactggttcaat3′

XIAP Sense 5′ggccagactatgcccattta3′

Antisense 5′cgaagaagcagttgggaaa3′

PDGFR Sense 5′ctctgacggccatgagtaca3′

Antisense 5′catgatcttcagctccgaca3′

β-Actin Sense 5′gtcgtaccactggcattgt3′

Antisense 5′cagctgtggtggtgaagct3′

### cDNA microarray analysis

We used PI3K-Akt pathway finder RT2 Profiler PCR Array (SuperArray Biosciences, Frederick, MD) because of its advantage of real-time PCR performance combined with the ability of microarrays to detect the expression of many genes simultaneously. Each array contains a panel of 96 primer sets of 84 relevant, pathway-focused genes, plus five housekeeping genes and three RNA and PCR quality controls. Real-time PCR was carried out under the following conditions: one cycle of 95°C for 10 min, 40 cycles of 95°C for 15 sec and 60°C for 1 min. Data were exported to Excel files and analyzed using SuperArray RT^2^ Profiler PCR Array Data Analysis Template (v3.0). Relative gene expression levels were calculated based on the ratio of the mean of housekeeping signals of all experiments. The formula used to calculate the relative gene expression level (2 ^∧^ (-Δ Ct)) in the “Results” worksheet is: Δ Ct  =  Ct (GOI) – avg. (Ct (HKG)), where GOI is each gene of interest, and HKG are the housekeeping genes chosen for the “Sample-Control Gene” worksheet. Scatter plots were made from normalized signals. Changes in gene expression were illustrated as a fold increase/decrease. The cut-off induction determining expression was 2.0 or −2.0 fold changes. Genes, which met these criteria, were considered to be upregulated or downregulated. We performed these experiments in duplicate.

RETRACTED

### Immunoblot analysis of proteins

Single and co-cultures of glioma cells or nude mice brain tissues were harvested and homogenized in four volumes of homogenization buffer (pH 7.4; 250 mM sucrose, 10 mM HEPES, 10 mM Tris-HCl, 10 mM KCl, 1% NP-40, 1 mM NaF, 1 mM Na_3_VO_4_, 1 mM EDTA, 1 mM DTT, 0.5 mM PMSF plus protease inhibitors: 1 µg/mL pepstatin, 10 µg/mL leupeptin and 10 µg/mL aprotinin) using a Teflon-fitted glass homogenizer. The homogenate was centrifuged at 20,000 *g* for 15 min at 4°C, and the protein levels in the supernatant were determined using the BCA assay (Pierce, Rockford, IL). Samples (40–50 µg of total protein/well) were subjected to 10–14% SDS-PAGE and transferred onto nitrocellulose membranes. The following antibodies were used for Western blot analysis: mouse anti-PTEN (1∶200; Santa Cruz Biotechnology Inc, Santa Cruz, CA), mouse anti-Fak (1∶500; Santa Cruz Biotechnology Inc), goat PI3K (1∶500; Santa Cruz Biotechnology Inc.), mouse anti-XIAP (1∶5000; BD Biosciences, Franklin Lakes, New Jersey), rabbit anti-AKT (1∶1000; Cell Signaling Technology), mouse anti-phospho-AKT (Ser^473^) (1∶1000; Cell Signaling Technology) mouse anti-Rho-A (1∶200; Santa Cruz Biotechnology Inc), rabbit anti-CDC42 [Phospho-Rac1/cdc42 (Ser^71^) antibody (1∶1000; Cell Signaling Technology)], mouse anti-PDGFR (1∶1000; Cell Signaling Technology), and mouse anti-RAC1(1∶1000; BD Biosciences). The membranes were blocked with 5% nonfat skim milk in PBS for 1 h at room temperature and then incubated with primary antibodies overnight at 4°C. The membranes were then processed with horse-radish peroxidase (HRP)-conjugated secondary antibodies. Immunoreactive bands were visualized using chemiluminescence ECL Western blotting detection reagents (Amersham, Piscataway, NJ). Immunoblots were stripped and re-developed with GAPDH antibody [mouse anti-GAPDH (1∶1000; Novus Biologicals, Littleton, CO)] to ensure equal loading levels. Experiments were performed in triplicates. Values for treated and untreated samples were compared using one-way ANOVA. A *p* value of <0.05 was considered significant.

RETRACTED

### Intracranial tumor growth

The Institutional Animal Care and Use Committee of the University of Illinois College of Medicine at Peoria, Peoria, IL, USA approved all surgical interventions and post-operative animal care. U251 (1×10^6^ cells) and 5310 (8×10^5^ cells) tumor cells were intracerebrally injected into the right side of the brains of nude mice, as described previously [57]. Seven days after tumor implantation, the mice were injected with hUCBSC near the left side of the brain. The ratio of the hUCBSC to cancer cells was maintained at 1∶4. Three weeks after tumor inoculation, six mice from each group were sacrificed by cardiac perfusion with 4% formaldehyde in PBS, their brains were removed, and paraffin sections were prepared. Sections were stained with H&E to visualize tumor cells and to examine tumor volume. The sections were blind reviewed by a neuropathologist and scored semiquantitatively for tumor size. Whole-mount images of brains were also taken to determine infiltrative tumor morphology. The average tumor area per section integrated to the number of sections where the tumor was visible was used to calculate tumor volume; tumor volumes were compared between controls and treated groups. RT-PCR was done on fresh brain tissue for FAK, PTEN, XIAP, PDGFR and β-actin.

### Immunohistochemical analysis

Brains of control and hUCBSC-treated mice brains were fixed in formaldehyde and embedded in paraffin as per standard protocols. Sections were deparaffinized as per standard protocol. Sections were blocked in 1% BSA in PBS for 1 h, and the sections were subsequently transferred to primary antibody diluted in 1% BSA in PBS (1∶100). Sections were allowed to incubate in the primary antibody solution overnight at 4°C in a humidified chamber. Sections were then washed in 1% BSA in PBS, incubated with the appropriate secondary antibody for 1 h and visualized using a confocal microscope. Transmitted light images were obtained after H&E staining as per standard protocol to visualize the morphology of the sections. For immunofluorescence, sections were treated with primary antibodies overnight at 4°C and then treated with appropriate Alexa flour secondary antibodies at room temperature for 1 h. Negative controls were maintained either without primary antibody or using IgG.

RETRACTED

### Statistical analysis

Quantitative data from cell counts, Western blot analysis, and other assays were evaluated for statistical significance using one-way analysis of variance (ANOVA). Data for each treatment group were represented as mean ± SEM and compared with other groups for significance by one-way ANOVA followed by Bonferroni's post hoc test (multiple comparison tests) using Graph Pad Prism version 3.02, a statistical software package. Results were considered statistically significant at a *p* value less than 0.05.

## Supporting Information

Figure S1 Spheroid migration in siPTEN transfected spheroids. (A) SNB19, U251, 4910 and 5310 cells were cultured in 96-well low attachment plates at a concentration of 5×10^4^ cells, and spheroids were allowed to grow for 24 h at 37°C with shaking at 40–60 rpm. The spheroids were then transferred to 48-well plates and were transfected with siPTEN for 60 h and then grown in conditioned medium from co-cultures and maintained for another 24–48 h. Spheroid migration was analyzed using a phase-contrast microscope. Scale bar = 1000 µm. (B) Quantitative analysis of spheroid migration from (A). Error bars indicate SEM. n = 3. Control = without any treatment and grown in glioma conditioned media; siPTEN = transfected with siPTEN and grown in glioma conditioned media; siPTEN + (Glioma cells +hUCBSC) =  transfected with siPTEN and grown in conditioned media from glioma cells + hUCBSC.
(7.50 MB TIF)

Figure S2 Monolayer wound-induced migration assay in conditioned media. A line was scratched with a 200-µm plastic pipette tip in SNB19, U251, 4910 and 5310 cultures. They were allowed to grow at 37°C in 5% CO_2_ atmosphere in conditioned media of glioma cells, hUCBSC and co-cultures. Every three hours, cells that had migrated to the wounded areas were photographed under a microscope for quantification of cell migration. Images are representative of three separate experiments. Scale bar  = 500 µm. (B) Quantitative analysis of wound-induced migration assay from (A). The results are presented as mean ± SEM of three experiments done in duplicate. CM  =  conditioned medium.
(7.93 MB TIF)
